# Analysis of Influencing Factors of Compliance with Non-Vitamin K Antagonist Oral Anticoagulant in Patients with Nonvalvular Atrial Fibrillation and Correlation with the Severity of Ischemic Stroke

**DOI:** 10.1155/2021/1021127

**Published:** 2021-10-19

**Authors:** Li Zhu, Xiaodan Zhang, Jing Yang

**Affiliations:** Clinical Nursing Teaching and Research Section, The Second Xiangya Hospital of Central South University, Changsha, Hunan 410011, China

## Abstract

Nonvalvular atrial fibrillation (NVAF) is associated with an increased risk of stroke and thrombus, and anticoagulant therapy is a key link in the prevention of stroke. At present, the anticoagulation rate of atrial fibrillation in China is low, and there are many factors affecting the adherence of patients with atrial fibrillation to anticoagulation. Non-vitamin K antagonist oral anticoagulants (NOACs) are anticoagulant with high application value due to their high safety and low risk of intracranial hemorrhage, stroke, and death. However, the compliance of NOACs is poor, and the current situation of anticoagulants in China is not optimistic. In this study, a total of 156 patients with NVAF who received NOAC anticoagulation therapy in our hospital from January 2018 to January 2019 were retrospectively analyzed. The results showed that education background, place of residence, number of complications, CHA2DS2-VASc score, and HAS-BLED score were independent influencing factors for NOACS compliance of NVAF patients. Also, the Pearson correlation analysis showed that there was a negative correlation (*r* = −0.465, *P* < 0.001) between NOAC compliance and severity of ischemic stroke in patients with NVAF. Therefore, clinical supervision and management of patients with NVAF after NOACs should be strengthened to improve the compliance of patients with NVAF after NOACs, reduce the damage of ischemic stroke, and improve their prognosis.

## 1. Introduction

Atrial fibrillation (AF) is an atrial rhythm with ineffective contractions and chaotic excitement caused by disorders of the heart's electrical system [1]. This is the most common persistent arrhythmia in clinical practice. Ischemic stroke is one of the most dangerous complications of AF. Epidemiological statistics show that the prevalence of AF in our country is 0.8%, and the incidence of subsequent ischemic stroke is up to 5%. [2]. Also, the annual incidence of ischemic stroke in patients with nonvalvular atrial fibrillation (NVAF) is 3–5 times that of patients with non-AF [2]. The non-vitamin K antagonist oral anticoagulants (NOACs) can effectively reduce the stroke risk of NVAF patients by 60%∼70% [3].

However, in the actual application of anticoagulation therapy, under the influence of individualized differences in dosages, cross reactions between medicines and foods, insufficient clinical anticoagulation therapy, and patients' lack of awareness of the necessity of anticoagulation, the overall treatment rate and medication compliance of NOAC anticoagulation in NVAF patients are not high [4, 5]. It largely increases the risk of ischemic stroke in patients with NVAF in China, and the severity of stroke and its recurrence rate are also affected [6]. Based on this, this research discusses the influencing factors of NOAC anticoagulation compliance in NVAF patients and their correlation with the severity of ischemic stroke. It is expected to provide relevant references for the improvement of compliance with NOAC anticoagulation therapy and the management of safety and effectiveness in clinical NVAF patients.

## 2. Materials and Methods

### 2.1. General Information

156 patients with NVAF who received NOAC anticoagulation therapy in our hospital from January 2018 to January 2019 were retrospectively analyzed. There were 87 males and 69 females, with an average age of (59.87 ± 11.64) years.

### 2.2. Inclusion Criteria

(i) All patients met the diagnostic criteria for NVAF in the 2017ACC Expert Consensus on Perioperative Anticoagulation Management Decisions in Patients with Nonvalvular Atrial Fibrillation [6]; (ii) the diagnostic criteria for patients with ischemic stroke were referred to the Chinese Guidelines for the Diagnosis and Treatment of Acute Ischemic Stroke (2018 edition); and (iii) patients who met the CHA2DS2-VASc (Including congestive heart failure/left ventricular dysfunction, hypertension, age ≥ 75 years, diabetes, history of stroke/TIA/thromboembolism, vascular disease, and female) and HAS-BLED (including hypertension, abnormal renal and liver function, stroke, bleeding, labile INRS, elderly, drugs, or alcohol) scoring criteria for NOACs anticoagulation [7].

### 2.3. Exclusion Criteria

(i) Accompanied by other diseases such as valvular disease and thromboembolic disease that require anticoagulation; (ii) pregnant and/or lactating women; (iii) patients with previous bleeding history; (iv) with other serious complications or important organ diseases; (v) patients with mental or consciousness disorders and communication difficulties; and (vi) patients who have joined other studies or received other anticoagulation therapy in recent 3 months.

### 2.4. Method

#### 2.4.1. Collecting the Baseline Information

All patients were followed up for 2 years, with an interval of 2 months in the first 6 months, an interval of 3 months in the next 6 months, and an interval of 4 months in the second year. Hospital review was the main method of follow-up.

The electronic medical records were used to collect baseline data on all patients, including gender, age, diploma, occupation, marriage, smoking history, drinking history, number of complications, number of drugs used for complications, CHA2DS2-VASc score, and HAS-BLED score. Also, personal health follow-up records were established according to the collected data.

#### 2.4.2. Survey of Compliance

Design of the medication compliance questionnaire: patient compliance was measured by the following four questions: (i) Can you take your medication as often as your doctor requires? (ii) Can you take the medication in the amount required by the doctor? (iii) Are you able to take your medication at the time and in the manner required by your doctor? (vi) Can you take your medication for a long period of time as required by your doctor? (v) Can you take your medication regularly according to your doctor's requirements? The options are “not at all,” “occasionally,” “basically,” and “completely,” respectively, 0∼3 points.

The total score ranges from 0 to 12 points. If the score is 12, the medication adherence is good. If the score is <12, the medication adherence is poor. In this study, the Cronbach's *α* coefficient of the questionnaire was 0.867, indicating good reliability.

#### 2.4.3. Investigation of Clinical End Points

At the last follow-up, the number of ischemic stroke, hemorrhagic events, and death cases in the good compliance group and poor compliance group was counted.

#### 2.4.4. Survey of Ischemic Stroke Severity

The severity of stroke in all patients with ischemic stroke was assessed using the NIH Stroke Scale (NIHSS) [8]. The full score of the NIHSS scale was 42; a score of 0-1 was classified as normal, 1∼4 as mild stroke/minor stroke, 5–15 as moderate stroke, 16–20 as moderate severe stroke, and 21∼42 as severe stroke.

### 2.5. Statistical Methods

All data were processed with SPSS 22.0 statistical software, and GraghPad prism 8 was used to make statistical graphs. Measurement data are expressed as mean ± standard deviation ($\bar{x}\pm s$), an independent-sample *t*-test is used for comparison between groups, count data are expressed as [*n* (%)], and the chi-square (*χ*^2^) test is performed. Factors significant in univariate analysis were subjected to multiple logistic regression model analysis. Correlation analysis was performed by Pearson correlation analysis. The difference is statistically significant when *P* < 0.05.

## 3. Results

### 3.1. Baseline Data and Compliance Scores of Follow-Up Patients

A total of 156 patients were followed up, and there were 8 cases of lost contact and 2 cases of death due to various reasons during the follow-up period. The actual number of effective cases during the follow-up period was 146, and the effective rate was 93.6%. The compliance score of 146 patients was (10.5 ± 1.4) points, among which 59 patients (40.4%) were in the good compliance group and 87 patients (59.6%) were in the poor compliance group (Table 1).

### 3.2. Univariate Analysis of Influencing Compliance with NOACs

Univariate analysis showed that age, educational background, place of residence, number of complications, CHA2DS2-VASc score, and HA-BLED score were the influencing factors for NOAC compliance of NVAF patients (*P* < 0.05) (Table 2).

### 3.3. Multivariate Analysis of Influencing Compliance with NOACs

The compliance was taken as the dependent variable, and the factors with significant differences in Table 2 were taken as independent variables into the logistic regression model. The assignments of the dependent variables and independent variables are shown in Table 3.

Education background, place of residence, number of complications, CHA2DS2-VASc score, and HAS-BLED score were independent influencing factors for oral NOACs compliance of NVAF patients (Table 4).

### 3.4. Comparison Scores of Clinical End Points between the Two Groups

The incidence of ischemic stroke in the good compliance group (5.1%) was lower than that in the poor compliance group (71.2%), and the difference was significant (*P* < 0.05). But, there was no significant difference in the incidence of hemorrhagic events between the two groups (*P* > 0.05). Among the patients who died, 2 patients in the poor compliance group died of stroke, while the remaining patients died of nonthromboembolism and hemorrhagic events (Table 5).

### 3.5. Correlation between NOAC Compliance and Severity of Ischemic Stroke

The types of stroke that occurred in the 3 patients in the good adherence group were all minor/minor stroke, and the types of stroke that occurred in the 12 patients in the poor adherence group were all moderate and major stroke (Table 6).

Pearson correlation analysis showed that there was a negative correlation (*r* = −0.791, *P* < 0.001) between NOAC compliance and severity of ischemic stroke in patients with NVAF (Figure 1).

## 4. Discussion

As a member of the cardiovascular epidemic in the 21st century, NVAF has become a major public health problem threatening the safety of citizens [9]. It occurs mainly in the middle-aged and elderly people with organic heart disease, and the prevalence was increased with age. The most serious complication after NVAF is thromboembolic events such as stroke [10]. According to statistics, about 13∼26% of ischemic strokes are directly associated with NVAF. Also, in patients of advanced age >80 years, AF is more a high-risk influential cause of concurrent ischemic stroke [11].

At present, NOACs are an approved treatment for thromboembolic disease in multiple clinical indications [12]. However, the investigation showed that the drug intake rate of patients with NVAF in China was extremely low, and the high prevalence of stroke and low rate of anticoagulant therapy have become the new features of atrial fibrillation patients in China [13].

With the wide application of the risk stratification and scoring tools for atrial fibrillation thrombosis and bleeding, such as CHA2DS2-VASc and HAS-BLED, clinical practice HAS-BLED found that it is of certain value to identify the risk of ischemic stroke and hemorrhagic transformation in NVAF patients before NOACs. It is not only beneficial to the correction of adverse events of NOACs but also enhances the confidence of clinical use of NOACs to a certain extent. In our study, 156 patients with NVAF who received NOACs in our institution were followed up for 2 years. The results showed that 87 patients (59.59%) were in the poor compliance.

Multiple logistic regression analysis was further used to confirm that education background, place of residence, number of complications, CHA2DS2-VASc score, and HA-BLED score were independent influencing factors for NOAC compliance of NVAF patients. The reasons include many aspects. First of all, in terms of educational background, patients with higher educational level have a higher understanding of NOACs and the individualized medication, so their subjective initiative of anticoagulation is also greater [14]. Secondly, compared with rural areas where communication and medical equipment are not well established, urban residents may have more advantages in regular monitoring, physician-patient interactions, and the popularization of relevant knowledge [15]. Thirdly, in terms of the number of complications, most patients with NVAF are complicated with basic diseases such as three highs, cardiovascular and cerebrovascular diseases, and liver and kidney diseases, which had higher variable in individuals, and a large impact on the blood concentration after treatment, and some patients may stop taking drugs or change medicines halfway, leading to a high probability of stopping medication or changing medication midway. At last, in terms of CHA2DS2-VASc and HAS-BLED score, patients with CHA2DS2-VASc score ≥2/3 (male/female) and HAS-BLED score ≥3 may be more aware of taking medicine due to the fear of discovering hemorrhagic conversion events under the crisis of high stroke risk [16].

In our study, the incidence of ischemic stroke in the good compliance group was lower than that in the poor compliance group, and the stroke degree of the 3 patients in the good compliance group was lower than that of the 12 patients in the poor compliance group. Moreover, Pearson correlation analysis showed that the compliance of NOACs in NVAF patients was negatively correlated with the severity of ischemic stroke [17]. These indicate that active and effective treatment with NOACs is an independent protective factor for effectively reducing the severity of ischemic stroke [18].

Some studies have pointed out the risk of bleeding rises accordingly when NOACs benefit [19]. In addition, due to differences in race, genetics, weight, and dietary structure, the hemorrhagic events in Chinese patients will increase. However, in practice, the benefits of NOAC therapy far outweigh the risks provided that the relevant guidelines are strictly followed, indications are properly mastered, embolism and bleeding risks are dynamically assessed, and coagulation function is closely monitored [20].

Notably, there was no significant difference in the incidence of hemorrhagic events between the good compliance group and the poor compliance group in our study. Possible reasons for this were the limited sample size and wide variation in age distribution in our study, and the sample subjects were not limited to elderly patients as in previous studies, which may have an impact on the results [21].

In conclusion, a variety of factors lead to the poor adherence of NOACs in NVAF patients. Therefore, clinical supervision and management of patients with NVAF after NOACs should be strengthened to improve the compliance of patients with NVAF after NOACs, reduce damage of ischemic stroke, and improve their prognosis.

## Figures and Tables

**Figure 1:** Correlation between NOAC compliance and severity of ischemic stroke. There was a negative correlation (*r* = −0.465, *P* < 0.001) between NOAC compliance and severity of ischemic stroke in patients with NVAF.

**Table 1:** Baseline information and the compliance scores of 146 follow-up patients (*n*, $\bar{x}\pm s$).

Clinical information	Baseline information situation
Gender	85 males (58.2%), 61 females (41.8%)
Age	53 patients with age <65 years (36.3%), 93 patients with age ≥65 years (63.7%)
Educational background	46 patients (31.5%) with no educational background/primary school, 58 patients (39.7%) with middle school/high school, and 42 cases (28.8%) with university or above
Place of residence	67 patients (45.9%) in rural areas and 79 patients (54.1%) in cities and towns
Marriage situation	69 patients were unmarried/widowed (47.3%), and 77 patients were married (52.7%)
Smoking history	51 patients (34.9%) had smoking history, 95 patients (65.1%) had no smoking history
Drinking history	56 patients (38.4%) had a history of drinking alcohol, 90 patients (61.6%) had no history of drinking alcohol.
Number of complications	0∼6 (2.9 ± 1.6) species
Number of concomitant medications	0∼8 (4.1 ± 2.1) species
CHA_2_DS_2_-VASc score	45 patients (30.8%) with scores <2/3 (male/female) and 101 patients (69.2%) with scores ≥2/3 (male/female)
HAS-BLED score	77 patients (52.7%) with score <3 and 69 patients (47.3%) with score ≥3
Compliance	(10.5 ± 1.4) points, good compliance in 59 patients (40.4%), poor compliance in 87 patients (59.6%)

**Table 2:** Univariate analysis of influencing compliance with NOACs (*n*, %, $\bar{x}\pm s$).

Clinical information	Good compliance group (*n* = 59)	Poor compliance group (*n* = 87)	*χ* ^2^/*t*	*P*
*Gender*				
Male	35 (59.3)	50 (57.5)	0.050	0.824
Female	24 (40.7)	37 (42.5)		

*Age*				
<65 years	41 (69.5)	40 (75.5)	7.870	0.001
≥65 years	18 (30.5)	47 (72.3)		

*Educational background*				
No educational background/primary school	28 (47.5)	18 (20.7)	16.350	≤0.001
Middle school/high school	18 (30.5)	40 (46.0)		
University or above	9 (15.3)	33 (37.9)		

*Place of residence*				
Rural area	49 (83.1)	18 (20.7)	55.062	≤0.001
Cities and towns	10 (16.9)	69 (79.3)		

*Marriage situation*				
Unmarried/widowed	36 (61.0)	33 (37.93)	7.518	0.006
Married	23 (29.87)	54 (70.13)		

*Smoking history*				
Yes	25 (42.4)	26 (29.9)	2.412	0.120
No	34 (57.6)	61 (70.1)		

*Drinking history*				
Yes	18 (30.5)	33 (37.9)	0.852	0.356
No	41 (69.5)	54 (62.1)		
Number of complications	2.6 ± 1.4	3.1 ± 0.9	2.627	0.012
Number of concomitant medications	4.3 ± 2.1	4.6 ± 2.2	0.823	0.412

*CHA*_2_ *DS*_2_ *-VASc score*				
<2/3 (male/female)	40 (67.80)	5 (5.75)	63.484	≤0.001
≥2/3 (male/female)	19 (32.20)	82 (94.25)		

*HAS-BLED score*				
<3 score	51 (86.44)	16 (18.39)	49.313	≤0.001
≥3 score	8 (13.56)	51 (58.62)		

**Table 3:** Variable assignment for multivariate analysis of influencing compliance with NOACs.

Variable	The assignment
*Dependent variable*	
Compliance	0 = good, 1 = poor
*Independent variables*	
Age	<60 years = 0, ≥60 years = 1
Marriage situation	Married = 0, unmarried/widowed = 1
Educational background	University or above = 0, middle school/high school = 1, no educational background/primary school = 2
Place of residence	Cities and towns = 0, rural area = 1
Number of complications	Enter the actual value
CHA_2_DS_2_-VASc score	≥2/3 (male/female) = 0, <2/3 (male/female) = 1
HAS-BLED score	≥3 score = 0, <3 score = 1

**Table 4:** Multivariate analysis of influencing compliance with NOACs.

Factors	*β*	SE	Wald	*P*	OR (95% CI)
Age ≥ 60 years	0.943	1.117	4.297	0.174	3.116 (0.561∼1.209)
Unmarried/widowed	1.165	2.545	4.436	0.098	1.765 (0.361∼1.935)

*Educational background*					
No educational background/primary school	5.112	1.628	9.817	0.007	166.861 (6.796∼4094.401)
Middle school/high school	3.290	1.432	5.254	0.027	26.983 (1.610∼451.128)

*Place of residence*					
Rural area	1.566	0.742	4.579	0.041	1.342 (0.571∼0.478)
Number of complications	0.928	0.454	4.136	0.047	2.538 (1.030∼6.244)

*CHA*_2_ *DS*_2_ *-VASc score*					
<2/3 (male/female)	2.211	0.982	5.004	0.029	0.106 (0.012∼0.756)

*HAS-BLED score*					
≥3 score	2.786	1.247	5.132	0.028	12.431 (0.964∼38.657)

**Table 5:** Comparison of clinical end points between the two groups (*n*, %).

Group	Ischemic stroke	Hemorrhagic events
Good compliance group (*n* = 59)	3 (5.1)	6 (10.2)
Poor compliance group (*n* = 87)	15 (17.2)	10 (11.5)
*χ* ^2^	4.807	0.063
*P*	0.028	0.801

**Table 6:** The compliance scores and NIHSS score of 15 patients with ischemic stroke (cases, points).

Group	Number	Compliance scores	NIHSS score
Good compliance group (*n* = 3)	7	12.0	3
	26	12.0	4
	69	12.0	2

Poor compliance group (*n* = 12)	4	9.3	31
	11	4.8	6
	28	10.5	22
	43	10.8	8
	47	11.0	15
	61	10.5	9
	70	10	23
	77	9.7	14
	85	4	19
	94	6.3	17
	97	5.5	24
	109	6.7	21

Note: a score of 0-1 was classified as normal, 1–4 as mild stroke/minor stroke, 5–15 as moderate stroke, 16–20 as moderate severe stroke, and 21–42 as severe stroke.

## Data Availability

The data used and analyzed during the current study are available from all the authors.
